RETRACTED

# MCCK1 enhances the anticancer effect of temozolomide in attenuating the invasion, migration and epithelial‐mesenchymal transition of glioblastoma cells in vitro and in vivo

**DOI:** 10.1002/cam4.1951

**Published:** 2019-01-18

**Authors:** Tie Liu, Anqi Li, Yulun Xu, Yu Xin

**Affiliations:** ^1^ Department of Neurosurgery Beijing Tiantan Hospital, Capital Medical University Beijing China

**Keywords:** epithelial‐mesenchymal transition, glioblastoma therapy, IKKε inhibitor, MCCK1, temozolomide

## Abstract

Chemotherapy with temozolomide (TMZ) is the traditional treatment for glioblastoma (GBM). Nevertheless, majority of GBM patients have recurrence from resistance to the chemotherapy. Herein, we examined combinational effects of MCCK1 (a specific and effective IKKε inhibitor) with TMZ in GBM U251MG and U‐87MG cell lines as well as U251MG xenograft models to overcome the therapeutic limitation of chemotherapy for GBM. Although MCCK1 alone showed inhibitory effects on in vitro proliferation, migration, invasion, and EMT of U251MG and U‐87MG cells, combination of MCCK1 and TMZ showed enhanced inhibitory effects. In the U251MG GBM xenograft models, MCCK1 showed synergistic therapeutic effects in combination with TMZ to reduce tumor volumes significantly. These data indicated that MCCK1 could be a candidate sensitizer to potentiate therapeutic effects of conventional cytotoxic treatment for GBM.

## 1 INTRODUCTION

Glioblastoma (GBM) is one of the most malignant and aggressive form of primary brain tumors.^1^ The clinical application of alkylating agent temozolomide (TMZ) is the biggest highlight of malignant GBM chemotherapy in nearly 10 years, and TMZ combined with radiotherapy has become the standard treatment for newly diagnosed GBM.^2^

Inhibitor of nuclear factor kappa‐B kinase subunit epsilon (IKKε, also called IKBKE) is a noncanonical member of the IκB kinase (IKK) family containing a series of serine/threonine kinases that include IKKα, IKKβ, TBK1, and the adaptor protein IKKγ.^3^, ^4^ It is worth noting that IKKε has been identified as an oncogenic protein in Ref. 5. IKKε was found to be upregulated aberrantly in breast cancer,^6^ ovarian cancer,^7^ and GBM.^3^, ^8^, ^9^ Therefore, IKKε inhibition is a desirable GBM therapeutic strategy as evidenced by abundance of researches.^10^, ^11^, ^12^ For example, Liu *et al *reported that a selective inhibitor of IKKε (Amlexanox) had anticancer effect in human GBM cell lines.^5^ Another study showed that IKKε silence contributed to proliferation‐ and invasion‐inhibition of GBM cells.^13^ Collectively, these data strongly support the role of IKKε in tumorigenesis.

So far, only a few small molecular inhibitors of IKKε are available. Bx‐795 was the first IKK active inhibitor on the market, which inhibits TBK1 and IKKε in vitro at the level of nmol concentration.^14^ However, the poor specificity of Bx‐795 limits the application. Bx‐795 was originally developed as an inhibitor of 3‐phosphoinositol dependent protein kinase 1 and was found to inhibit IKKε later.^15^ Moreover, Bx‐795 showed off‐target effect on several other kinases, including JNK and p38MAP kinases.^16^ MRT67307 is an improved version of Bx‐795 without inhibition on JNK or p38MAP kinases. However, MRT67307 still interferes with the activities of TBK1 and PDK1.^16^ Therefore, it is necessary to develop a specific and effective IKKε inhibitor.^17^

RETRACTED

In our previous study (in press), we screened a specific and effective IKKε inhibitor, named MCCK1 (Malachite Green Oxalate), which was found to inhibit IKKε and the downstream factors such as IkBa, p65, and IRF3. MCCK1 was identified to reduce the resistance of GBM cells to TMZ, and significantly enhance the efficiency of TMZ to inhibit cell proliferation and induce apoptosis. In the present study, we aim to explore the effect of MCCK1 on invasion, migration, and epithelial‐mesenchymal transition (EMT) of GBM U251MG and U‐87MG. Meanwhile, the synergistic effects of MCCK1 and TMZ were studied.

## 2 METHODS AND MATERIALS

### 2.1 Cell culture and reagents

The human GBM cell lines U‐251MG and U‐87MG (American Type Culture Collection) were separately cultured in Dulbecco's modified essential medium (DMEM; Gibco, Rockville, MD) and Eagle's Minimum Essential Medium (EMEM; Gibco) supplemented with 10% fetal bovine serum (FBS; Gibco), penicillin (100 units/mL; Gibco), and streptomycin (100 g/mL; Gibco). These cells were maintained at 37°C in an incubator with 5% CO_2_. MCCK1 was purchased from Sigma‐Aldrich and dissolved in 10% dimethyl sulphoxide (DMSO; Sigma‐Aldrich) to create a stock solution (100 mg/mL). Working concentrations were freshly prepared daily by diluting the stock with PBS. TMZ was purchased from Sigma‐Aldrich and dissolved in 10% DMSO (Sigma‐Aldrich) to create a stock solution (TMZ: 100 mg/mL).

### 2.2 Cells and animals grouping

U‐251MG and U‐87MG cells were treated with NC (Ctrl), 2.5 μmol/L MCCK1 (MCCK1), 100 μmol/L TMZ (TMZ), and MCCK1 (2.5 μmol/L) + TMZ (100 μmol/L). The orthotopic xenograft models were established using female BALB/c athymic nude mice (6‐week‐old), and divided into four group with treatment of (a) cTRL (normal saline, every day from 1 day after tumor cell implantation), (b) MCCK1 (15 mg/kg, every day from 1 day after tumor cell implantation), (c) TMZ (2 mg/kg, every day from 1 day after tumor cell implantation), or (d) MCCK1 (15 mg/kg)+ TMZ (2 mg/kg).

RETRACTED

### 2.3 Cell counting kit‐8 cell viability assay

Cell counting kit‐8 (CCK‐8) assay was performed to test cell toxicity of MCCK1 and proliferation of U‐251MG and U‐87MG cells in this study. For toxicity test, the U‐251MG and U‐87MG cells treated with MCCK1 (0, 0.1, 0.25, 0.5, 1.0, 2.5, 5, 10, 25, 50, 100 μmol/L) for 48 hours, cells were collected to detect the OD490. For proliferation determination, U‐251MG and U‐87MG cells were pretreated with NC, 2.5 μmol/L MCCK1, 100 μmol/L TMZ and MCCK1 (2.5 μmol/L) + TMZ (100 μmol/L) for 24 hours, then cells were trypsinized and seeded into 96‐well plates at a density of 1.5 × 10^3^ cells in 200 μL of full medium each well. After this, the plate was incubated at 37°C with 5% CO_2_. CCK‐8 assay was performed using CCK‐8 kit as the manufacturer's instructions for the next continuous 4 days. Absorbance at 490 nm (OD490) was detected by using a microplate reader (BioTek Instruments, Inc, Winooski, VT).

### 2.4 Hoechst 33342 staining

U‐251MG and U‐87MG cells were detached from the culture dish and resuspended in DMEM medium containing 2% FBS at a density of 1 × 10^6^ cells/mL. Then, cells were incubated with Hoechst 33342 staining solution (Sigma‐Aldrich) for 60 minutes at 37°C according to the manufacturer's instruction. Finally, cells were observed under a fluorescence microscopy. Apoptotic cell death was determined by counting the number of cells with condensed nuclei in six randomly selected areas.

### 2.5 Western blotting analysis

U‐251MG and U‐87MG cells were treated with MCCK1 (2.5 μmol/L) or TMZ (100 μmol/L) for 48 hours. Cells were collected and tumors tissues were homogenized. Protein was extracted with RIPA lysis buffer adding cocktail (Sigma‐Aldrich) and phenylmethanesulfonyl fluoride (PMSF; Sigma‐Aldrich). Equal amounts of protein (40 µg) were resolved on (6%‐12%) SDS‐PAGE, transferred onto PVDF membranes (Millipore, Billerica, MA), probed with primary antibodies. Antibodies were as follows: antiVimentin (Abcam, Cambridge, MA), antiGAPDH (Abcam), antiKi67 (Abcam), antiCaspase‐3 (Abcam), antiVEGF (Abcam), antiMMP‐14 (Abcam), antiEcadherin (Abcam), antiTwist1 (Abcam), antizeb1 (Abcam), antizeb2 (Abcam), antiNcadherin (Abcam), antiSnail1 (Cell Signaling Technology, Beverly, MA). After incubation with the proper horseradish peroxidase (HRP)‐conjugated secondary antibody (Santa Cruz Biotechnology, Santa Cruz, CA), proteins were detected using a ChemiDoc xRS imaging system and Quantity One analysis software (Bio‐Rad Laboratories, San Francisco, CA). Antibodies were visualized the Amersham ECL Prime Western Blotting Detection Reagent (GE Healthcare, UK).

### 2.6 Xenograft tumor model

For efficacy test of MCCK1 combined TMZ in vivo, we established the orthotopic xenograft models by intracranial injection using 6‐week‐old female athymic nude mice. To establish the orthotopic xenograft models, U‐251MG cells (2 × 10^5^/5 L Hank's balanced salt solution [HBSS], Gibco) were stereotypically injected into the left striata of mice. Animals were divided into four groups: NC (cTRL), MCCK1, TMZ, MCCK1+TMZ. Each group had eight mice, and mice were medicated by MCCK1 (5 mg/kg for every day via per oral) at 1 day after tumor cells injection. TMZ (2 mg/kg × 5 via per oral) 30 days after tumor cells injection. All animals were sacrificed at 30 days, median survival of the orthotopic xenograft model using U‐251MG a cells. Tumor diameter was measured using vernier caliper, and tumor volume determined by calculating the volume of an ellipsoid using the formula: (length × width^2^ × 0.5).

RETRACTED

### 2.7 TUNEL

Terminal deoxynucleotidyl transferase‐mediated dUTP‐biotin nick end labeling (TUNEL) staining was performed to detect apoptosis in situ cell death according to the manufacturer's instructions (TUNEL Apoptosis detection kit: UPSTATE, Lake Placid, NY). TUNEL‐positive cells displayed brown staining within the nucleus of apoptotic cells. The extent of apoptosis was calculated and expressed as a number of TUNEL‐positive cells from the same field.

### 2.8 Immunohistochemistry

The paraffin‐embedded tumor sections were stained for antiKi67, antiCaspase‐3, and antiVEGF (Abcam, Cambridge, UK). Sections (2 μm) were deparaffinized and pretreated with citrate buffer using a heat‐induced epitope retrieval protocol. Endogenous peroxidase was blocked with 20% hydrogen peroxide for 15 minutes at room temperature followed by incubation with antiKi67, antiCaspase‐3, and antiVEGF for 30 minutes, respectively. A biotinylated goat antimouse immunoglobulin G secondary antibody (Dako, Denmark) was then applied to each slide for 30 minutes. After washing in Tris‐hydrochloric acid buffer (TBS), the slides were incubated with peroxidase‐conjugated streptavidin complex reagent (Dako) and developed with 3,3′‐diaminobenzidine for 5 minutes. The slides were counterstained and dehydrated.

### 2.9 Statistics analysis

The results were expressed as mean values ± standard deviation (SD) or standard effort (SE). Statistical comparisons were analyzed by one‐way analysis of variance (ANOVA) followed by the least significant difference (LSD) test. A significant level of <0.05 was used for all tests. SPSS‐PASW statics software version 18.0 was used for all the statistical analyses.

## 3 RESULTS

### 3.1 MCCK1 enhanced the proliferation‐inhibiting and apoptosis‐promoting effect of TMZ

To clarify the influence of MCCK1 on GBM cells, we first performed a CCK‐8 assay using U‐251MG GBM cells treated with MCCK1 at concentrations of 0‐100 μmol/L for 24 hours, respectively. The result (Additional file 1) showed that MCCK1 exerted an inhibitory effect on GBM cells in a dose‐dependent manner (*P* < 0.05; compared to 0 hour). The concentration of inhibited cell viability was at 2.5 μmol/L in U‐251MG cells. In addition, treatment with MCCK1 at 2.5 μmol/L did not induce significant cytotoxicity of U‐251MG cells. Thus, 2.5 μmol/L of MCCK1 was used for subsequent experiments. About 100 μmol/L TMZ was used as previous study.^18^ As shown in Figure 1A,B, both MCCK1 and TMZ suppressed the growth of U‐251MG and U‐87MG cells compared with the control (*P < *0.05). However, the combination of MCCK1 and TMZ enhanced the proliferation‐inhibiting effect compared with the TMZ group (*P < *0.05). As shown in Figure 1C‐H, both MCCK1 and TMZ promoted the apoptosis of U‐251MG and U‐87MG cells compared with the control (*P < *0.05). In addition, the combination of MCCK1 and TMZ enhanced the apoptosis‐promoting effect compared with the TMZ used alone at the same dose (*P <* 0.05). The present results were verified by western blot analysis of Ki67 and Caspase‐3 exhibited in Figure 1I,J. The relative expression of Ki67 was significantly reduced by MCCK1 and TMZ, and combination therapy (*P < *0.05), while the expression of caspase‐3 exhibited reversed results.

RETRACTED

**Figure 1:** MCCK1 enhanced the proliferation‐inhibiting and apoptosis‐promoting effect of TMZ. (A) U‐251MG and (B) U‐87MG cells were cultured in 96‐well plates and then treated with solvent only (Ctrl) or 100 μmol/L TMZ with 2.5 μmol/L MCCK1 for 48 h. OD490 of U‐251MG and U‐87MG cells were determined by CCK‐8. (C) Apoptosis of U‐251MG cells was detected by Hoechst 33258 staining. (D) The representative column diagrams showing results of apoptosis rate of U‐251MG cells. (E) Apoptosis of U‐87MG cells was detected by Hoechst 33258 staining. (F) The representative column diagrams showing results of apoptosis rate of U‐87MG cells. (G) Apoptosis of U‐87MG cells was detected by flow cytometry.(H) The representative column diagrams showing results of ratios of Q2 + Q4 in Figure 1G. (I) The protein expression was detected by western blot. GAPDH was used as the loading control. (J) The representative column diagrams showing results of relative protein expression. *P < 0.05, compared with Ctrl, *#P < *0.05, compared with TMZ. Data are mean ± SEM for the three replicates

### 3.2 MCCK1 enhanced the invasion‐inhibiting and migration‐inhibiting effect of TMZ

U‐251MG and U‐87MG cells were treated as previous described. Wound healing assay and transwell assay were carried out separately for migration and invasion testing. As shown in Figure 2A and C, both MCCK1 and TMZ suppressed the numbers of invasive U‐251MG and U‐87MG cells compared with the control (*P <* 0.05). Expectedly, the combination of MCCK1 and TMZ enhanced the invasion‐inhibiting effect compared with the TMZ group (*P < *0.05). Similarly, both MCCK1 and TMZ suppressed the wound closure rate of U‐251MG and U‐87MG cells compared with the control (*P < *0.05). Meanwhile, the combination of MCCK1 and TMZ enhanced the migration‐inhibiting effect compared with the TMZ used alone at the same dose (Figure 2B and D, *P <* 0.05). The expression of metastasis‐related maker VEGF and MMP‐14 were conducted by western blot assay, the result demonstrated that the relative expression of VEGF and MMP‐14 were significantly reduced by combination therapy compared with the TMZ used alone at the same dose (Figure 2E‐J, *P < *0.05).

RETRACTED

**Figure 2:** MCCK1 enhanced the invasion‐inhibiting and migration‐inhibiting effect of TMZ. A, Cell invasion of U‐251MG was analyzed by Transwell assay (magnification, ×400). B, Cell migration of U‐251MG was analyzed by wound healing assay. The upper figures showed the four groups of U‐251MG cells scraped by a pipette tip at zero time, wound width = a. The lower figures showed the morphology at 24 h, wound width = b. Wound closure rate = (a−b)/a*%, (magnification, ×200). C, Cell invasion of U‐87MG was analyzed by Transwell assay (magnification, ×400). D, Cell migration of U‐87MG was analyzed by wound healing assay. E, The protein expression was detected by western blot. GAPDH was used as the loading control. F‐G, The representative column diagrams showing results of relative protein expression. *P < 0.05, compared with Ctrl*, #P <* 0.05, compared with TMZ. Data are mean ± SEM for the three replicates

### 3.3 Combining MCCK1 and TMZ treatment reduced EMT of U‐251MG and U‐87MG cells

To clarify the mechanism of metastasis‐inhibiting effect of MCCK1 cooperating with TMZ, U‐251MG, and U‐87MG cells were treated as previous described and observed under a phase contrast microscope. As shown in Figure 3A, spindle‐shaped like cells were significantly reduced and flat cells were increased in MCCK1+TMZ group, this morphological feature indicated that cell adhesion was attenuated by combination therapy. We next detected the expression of EMT maker protein, including E‐cadherin, Twist1, zeb1, zeb2, N‐cadherin, Vimentin, and Snail. As a result, except E‐cadherin, the expression of Twist1, zeb1, zeb2, N‐cadherin, Vimentin, Snail were all inhibited by MCCK1, TMZ, or combination therapy (Figure 3B,C, *P < *0.05). Moreover, we checked the expression of Vimentin by immunofluorescence. Green fluorescence represented the existence of Vimentin. MCCK1 and TMZ combination therapy obviously reduced green fluorescence (Figure 3D,E*, P *< 0.05). These results indicated that combining MCCK1 and TMZ treatment significantly reduced EMT of U‐251MG and U‐87MG cells.

RETRACTED

**Figure 3:** Combining MCCK1 and TMZ treatment reversed EMT of GBM cells. A, Morphological changes in U‐251MG and U‐87MG cells (magnification, ×100). B, The protein expression was detected by western blot. GAPDH was used as the loading control. C, The representative column diagrams showing results of relative protein expression. D, Vimentin (green) in U‐251MG and U‐87MG cells was detected by immunocytochemistry. DAPI (blue) = nuclei. E, The representative column diagrams showing the Vimentin‐positive cells ratio. *P < 0.05, compared with Ctrl*, #P < *0.05, compared with TMZ. Data are mean ± SEM for the three replicates

### 3.4 MCCK1 enhanced the growth‐inhibiting effect of TMZ in U‐251MG and U‐87MG orthotopic xenograft models

We employed U‐251MG and U‐87MG orthotopic xenograft models to confirm the in vitro combinational treatment result of MCCK1 in vivo. Node mice were treated with NC (cTRL), MCCK1 (15 mg/kg BW), TMZ (2 mg/kg BW), or MCCK1 (15 mg/kg BW) + TMZ (2 mg/kg BW) combination. Tumor volume and survival were analyzed for 30 days after tumor cell implantation. At the 30th day, mice were sacrificed for immunohistochemistry, TUNEL, and western blot assay. As shown in Figure 4A, the combination treatment with MCCK1 and TMZ significantly decreased xenograft tumor volume, while the single treatments of MCCK1 or TMZ slightly decreased tumors size. In addition, combination therapy dramatically increased the survival of nude mice (Figure 4B). The TUNEL result combined with immunohistochemistry result demonstrated that combination treatment with MCCK1 and TMZ significantly promoted apoptosis of xenograft tumor cells, immunohistochemistry of Caspase‐3 confirmed the elevated apoptosis (Figure 4C,D). Meanwhile, the low expression of Ki67 and VEGF indicated a suppression of invasion and proliferation by combination of MCCK1 and TMZ (Figure 4E,F). The EMT markers were detected in tumor tissues (Figure 5). Combination therapy significantly increased the E‐cadherin level and reduced the Twist1, zeb1, zeb2, vimentin, N‐cadherin, and Snail level (*P < *0.05). The in vivo results were consistent with those in vitro*.*

**Figure 4:** MCCK1 enhanced the growth‐inhibiting effect of TMZ in vivo. A, Nude mice bearing subcutaneous xenograft GBMs were treated with cTRL, MCCK1, TMZ, and MCCK1+TMZ. The volume of tumor was determined every 5 days for 30 days. B, The survival of mice was determined every 3 days for 30 days. C, TUNEL assay was used to determine the apoptosis in MCCK1, TMZ, and combination therapy treated tumors compared with NC‐treated tumors (magnification, ×200). D, The representative column diagrams showing results of apoptosis rate. E, Immunohistochemistry analysis of expression of Ki67, Caspase‐3, and VEGF (magnification, ×200). F, The representative column diagrams showing results of positive cells (brown). *P < 0.05, compared with cTRL*, #P < *0.05, compared with TMZ. The results were analyzed by one‐way ANOVA followed by the least significant difference (LSD) test

**Figure 5:** MCCK1 enhanced the EMT‐inhibiting effect of TMZ in vivo. Western blot analysis showed that the protein expression of N‐cadherin, Vimentin, and Snail decreased, and the protein expression of E‐cadherin increased in tumors, especially in the MCCK1+ TMZ group. *P < 0.05, compared with cTRL*, #P < *0.05, compared with TMZ. Data are mean ± SEM for the three replicates

RETRACTED

## 4 DISCUSSION

Glioblastoma is a malignant tumor characterized by high proliferative and invasive capability.^19^ Meanwhile, GBM is one of the most resistant tumors to conventional chemotherapy, which results in poor survival from traditional surgical tumor resection supplemented with chemotherapy or radiotherapy.^20^, ^21^ To overcome the barrier, current studies concentrate on combinations with other agents and on development of novel molecular targeting agents.^22^, ^23^, ^24^ Recently, improvement of TMZ resistance on GMB was reported largely.^18^, ^25^, ^26^, ^27^ For example, a varies of microRNAs and agents were found to enhance the sensitivity of GBM to TMZ.^18^, ^25^, ^26^, ^27^ In present study, we confirmed that MCCK1 enhanced proliferation‐inhibiting and apoptosis‐promoting effects of TMZ. We also demonstrated that MCCK1 enhanced the antimigratory and antiinvasive effects of TMZ.

MCCK1 is an oxalate form of malachite green (MG) oxalate form. MG, as a triphenylmethane dye, is used to control parasitic infections in aquaculture. Though previous study demonstrated that treatment with MG does not reduce reproductive potential of zebrafish fish, MG was reported to be a teratogenic or carcinogenic compound.^28^ As far as I know, this is the first time we point out MG has the anticancer property. In the present study, we determined the toxicity of MCCK1 on U‐251MG (see Supporting Information). The treatment concentration more than 5 μmol/L of MCCK1 significantly reduced the cell viability*. *In vitro, treatment with doses (2.5 μmol/L) for 48 hours does not cause significant damage to U‐251MG cells, which suggests appropriate doses for studying in vitro experiments. We determined the influence of MCCK1 and TMZ on proliferation and apoptosis in U‐251MG and U‐87MG cells. In vivo, the decreased volume of xenograft tumor and increased the survival of xenograft tumor model mice confirmed the proliferation‐inhibiting effect of MCCK1. Collectedly, the results indicated that MCCK1 enhanced the proliferation‐inhibiting and apoptosis‐promoting effects of TMZ on U‐251MG and U‐87MG cells and xenograft tumor model mice.

RETRACTED

Epithelial‐mesenchymal transition is a reversible biological process involved in embryogenesis, tissue regeneration and cancer progression.^29^ In primary tumors, the decreased epithelial markers such as E‐cadherin and the increased mesenchymal markers including N‐cadherin, vimentin, and Snail can promote the tumor invasion and metastasis.^3^, ^30^ Whether EMT has a real association with malignant GBM invasion remains controversial.^31^ Previous studies highlighted numerous EMT markers that play an important role in GBM malignancy.^32^ Myung *et al* demonstrated that Snail promoted EMT, cell proliferation, migration, and invasion in GBM.^33^ In the present study, both MCCK1 and TMZ suppressed the EMT of GBM in vitro, evidenced by decreased E‐cadherin and increased N‐cadherin, vimentin, and Snail as well as the morphological change. Compared with single MCCK1 or TMZ, the stronger inhibitory effect on EMT was observed in MCCK1 and TMZ combination. Further, in vivo study showed that nude mice treated with either MCCK1/TMZ or combination therapy attenuated the EMT. Our study indicated that MCCK1 enhanced the anticancer effect of TMZ in attenuating the invasion, migration, and EMT of GBM cells in vitro and in vivo.

Since the mechanism of how MCCK1 regulated invasion, migration, and EMT is not studied, it is reasonable to speculated that MCCK1 played antiGBM role via targeting IKKε. As evidenced by our previous study (in press), MCCK1 is a specific and effective IKKε inhibitor. Pervious study showed that IKKε could regulate GBM cell proliferation, migration, and invasion abilities in vitro and in vivo via the Hippo pathway.^3^ The research also revealed that IKKε could accelerate EMT of GBM cells.^3^ Another IKKε selective inhibitor, amlexanox was reported to generate antitumor effects by disrupting the Hippo pathway in human GBM cell lines.^5^ We guess that MCCK1 may inhibit IKKε to play anticancer role, but the regulatory mechanism of MCCK1 need to be further explored.

In summary, as a selective IKKε inhibitor, MCCK1 is proved to enhance the anticancer effect of TMZ in attenuating the invasion, migration, and EMT of GBM cells in vitro and in vivo*.* MCCK1 has the potential to become a novel chemical for GBM therapy combined with TMZ.
